The article "Mechanical Stretch Promotes Macrophage Polarization and Inflammation via the RhoA-ROCK/NF-κB Pathway" was published in 2022. Journal: Biomed Res Int.

# Mechanical Stretch Promotes Macrophage Polarization and Inflammation via the RhoA-ROCK/NF-*κ*B Pathway

**DOI:** 10.1155/2022/6871269

**Published:** 2022-07-23

**Authors:** Peng-cheng Tu, Ya-lan Pan, Zhong-qing Liang, Guang-lu Yang, Cheng-jie Wu, Liang Zeng, Li-ning Wang, Jie Sun, Meng-min Liu, Yong-feng Yuan, Yang Guo, Yong Ma

**Affiliations:** ^1^Affiliated Hospital of Nanjing University of Chinese Medicine, Nanjing 210029, China; ^2^Laboratory of New Techniques of Restoration and Reconstruction of Orthopedics and Traumatology, Nanjing University of Chinese Medicine, Nanjing 210023, China; ^3^Nursing Institute of Integrated Chinese and Western Medicine, Nanjing University of Chinese Medicine, Nanjing 210029, China; ^4^School of Chinese Medicine, School of Integrated Chinese and Western Medicine, Nanjing University of Chinese Medicine, Nanjing, Jiangsu 210023, China

## Abstract

Macrophages play an essential role in the pathogenesis of most inflammatory diseases. Recent studies have shown that mechanical load can influence macrophage function, leading to excessive and uncontrolled inflammation and even systemic damage, including cardiovascular disease and knee osteoarthritis. However, the molecular mechanism remains unclear. In this study, murine RAW264.7 cells were treated with mechanical stretch (MS) using the Flexcell-5000T Tension System. The expression of inflammatory factors and cytokine release were measured by RT-qPCR, ELISA, and Western blotting. The protein expression of NF-*κ*B p65, I*κ*b-*α*, p-I*κ*b-*α*, RhoA, ROCK1, and ROCK2 was also detected by Western blotting. Then, Flow cytometry was used to detect the proportion of macrophage subsets. Meanwhile, Y-27632 dihydrochloride, a ROCK inhibitor, was added to knockdown ROCK signal transduction in cells. Our results demonstrated that MS upregulated mRNA expression and increased the secretion levels of proinflammatory factors iNOS, IL-1*β*, TNF-*α*, and IL-6. Additionally, MS significantly increased the proportion of CD11b+CD86+ and CD11b+CD206+ subsets in RAW264.7 macrophages. Furthermore, the protein expression of RhoA, ROCK1, ROCK2, NF-*κ*B p65, and I*κ*B-*α* increased in MS-treated RAW264.7 cells, as well as the IL-6 and iNOS. In contrast, ROCK inhibitor significantly blocked the activation of RhoA-ROCK and NF-*κ*B pathway, decreased the protein expression of IL-6 and iNOS, reduced the proportion of CD11b+CD86+ cells subpopulation, and increased the proportion of CD11b+CD206+ cell subpopulation after MS. These data indicate that mechanical stretch can regulate the RAW264.7 macrophage polarization and enhance inflammatory responses in vitro, which may contribute to activation the RhoA-ROCK/NF-*κ*B pathway.

The article "Mechanical Stretch Promotes Macrophage Polarization and Inflammation via the RhoA-ROCK/NF-κB Pathway" was published in 2022. Journal: Biomed Res Int.

## 1. Introduction

Inflammation is a defensive response to harmful stimuli, such as trauma and biological pathogen like bacteria and viruses [1]. However, uncontrolled inflammation can lead to local tissue injury or even systemic damage, including acute lung injury and osteoarthritis [2]. Macrophages, an important immunological cell, play a critical role in the most inflammatory processes, including innate immunity, antigen presentation, and immune regulation [3–5]. Faced with complex microenvironmental stimuli *in vivo*, macrophages can be triggered into two subtypes: classic M1-type and alternatively activated M2-type [6, 7]. M1-type macrophages, characterized by CD86 expression, can be activated by lipopolysaccharides (LPS) and interferon and secrete many proinflammatory factors, such as interleukin-1*β* (IL-1*β*) or inducible nitric oxide synthase (iNOS) [8]. Moreover, overactivation of NF-*κ*B promotes M1 macrophage polarization, leading to overwhelming uncontrolled inflammation and tissue damage [9]. M2-type macrophages, marked by CD206 expression, can be activated by IL-13 and IL-4, and secrete IL-10 and Arginase-1 to limit excessive inflammatory responses, which are related to tissue repair and angiogenesis [10, 11]. Therefore, sustained M1-type proinflammatory responses tend to disrupt the M1/M2 inflammatory balance, causing the activation of a large number of inflammatory cells and the overexpressed inflammatory chemokines, leading to the occurrence of inflammatory syndrome like rheumatoid arthritis [12]. In addition to the biological and chemical factors, mechanical stimulation can also regulate macrophage function and behavior. Mounting evidences show that mechanical stimulation contributes to pathophysiologic processes in diseases such as knee osteoarthritis [13], cardiac fibrosis [14], and cancer [15], where changes in the cellular mechanical microenvironment may be a key driver of specific cell behavior. Significant efforts have been made to elucidate the effect of mechanical microenvironmental cues on macrophages [16, 17]. Macrophages found in plaque areas of the coronary arteries in vivo, suffering from higher mechanical pressure than normal blood vessels, are involved in atherogenesis [18]. Atcha et al. [19] found that uniaxial stretch altered the macrophage morphology and activation responses via integrin CD11b and mechanosensitive ion channel Piezo1. Shan et al. [20] found that mechanical stretch can promote M1-type activation of macrophages by activating Focal Adhesion Kinase (FAK). However, more research is still needed to study the effects and mechanism of mechanical stimulation on macrophages.

Ras homolog gene family, member A (RhoA), and Rho-associated protein kinase (ROCK) are the major cytoskeletal regulatory factors. Overexpression of RhoA-ROCK is associated with macrophage proliferation, differentiation, [21–24], adhesion, migration, and infiltration of monocytes in the inflammatory process [25, 26]. Several reports have shown that RhoA-ROCK signaling pathway is involved in response to abnormal mechanical load through regulating the cell actin cytoskeleton and imbalance of *β*-catenin [18, 27]. These data indicate that RhoA-ROCK may play an important role in the polarity and functions of macrophage induced by mechanical stimuli. Therefore, this study is aimed at exploring the effects of mechanical stimulation on macrophage, RAW264.7 cells, and its involved signal pathway.

The article "Mechanical Stretch Promotes Macrophage Polarization and Inflammation via the RhoA-ROCK/NF-κB Pathway" was published in 2022. Journal: Biomed Res Int.

## 2. Materials and Methods

### 2.1. Cells and Reagents

Murine RAW264.7 cells were was obtained from Kaiji (Nanjing China). ELISA kits for IL-1*β*, TNF-*α*, and iNOS were purchased from Abbkine (USA). And ELISA kit for IL-6 was purchased from Fcmacs (Nanjing, China). FITC-CD11b, PE-CD86, and APC-CD206 antibody were obtained from BD Biosciences (USA); FITC-labeled phalloidin was obtained from Yeasen (Shanghan, China). Anti-mouse RhoA, ROCK, NF-*κ*B, I*κ*B, or p-I*κ*B antibodies were purchased from CST (USA), and anti-mouse GAPDH, iNOS, and IL-6 antibodies were purchased from Proteintech (Wuhan, China). Y-27632 dihydrochloride, a ROCK inhibitor, was obtained from Tocris Bioscience (USA).

### 2.2. Stretch Stress Intervention

RAW264.7 macrophages were plated on 6-well plates cultured with h-DMEM (BioInd, Israel), containing 100 U/ml penicillin-streptomycin and 10% fetal bovine serum (BioInd, Israel) at 37°C, 5% CO_2_. When cell density reached 60-70%, mechanical stretch was performed using the Flexcell-5000T Tension system [20, 28, 29] (0.5 Hz, rounds of pull 6 s-stop 6 s for 8 h at 0, 5, 10, and 15% elongation). In addition, Y-27632 dihydrochloride, a selective ROCK inhibitor, was added to the medium at 10 nM.

### 2.3. Morphological Observation

After mechanical stretch, macrophages in each group were collected and observed under a microscope. The supernatants were discarded, the cells were fixed with 4% paraformaldehyde for 25 minutes. The cells were then incubated at 5% Triton x-100 (Sigma, USA) for 10 minutes. Subsequently, the cells were incubated with FITC-labeled phalloidin solution in darkness at 25°C for 30 min. The cell morphology was observed by fluorescence microscope (Olympus, Japan) at 496 nm and 516 nm, respectively.

### 2.4. Determination of Cytokine Release in Culture Supernatant

After mechanical stretch, RAW264.7 macrophage culture medium was collected and the supernatant was centrifuged to determine the concentration of inflammation cytokines. TNF-*α*, iNOS, IL-1, and IL-6 in cell supernatants were detected by ELISA according to the manufacturers' instructions.

The article "Mechanical Stretch Promotes Macrophage Polarization and Inflammation via the RhoA-ROCK/NF-κB Pathway" was published in 2022. Journal: Biomed Res Int.

### 2.5. Flow Cytometry (FCM)

RAW264.7 macrophages were collected after mechanical stretch, washed, and centrifuged with cold buffer solution. The cells were resuspended with 5 *μ*l PE-CD86, 5 *μ*l FITC-CD11b, and 100 *μ*l combined buffer, respectively, and incubated for 30 min shielded from light. Then, the cells were fixed and permeabilized using Fixation & Permeabilization Kit (Fcmacs, Nanjing) according to the instructions. Subsequently, APC Rat anti-CD206 was added. After 15 min of incubation, the cells were washed and then analyzed by Amnis FlowSight flow cytometer (Merck Millipore, USA).

### 2.6. Quantitative Real-Time PCR (RT-qPCR)

The RNA Isolation Kit, PrimeScriptTM RT Master Mix, and TB Green™ Premix Ex Taq™ II kit were provided by Vazyme. Total RNA of RAW264.7 macrophages after mechanical stretch was extracted and then reversely transcribed into cDNA. RT-qPCR was performed using an Applied Biosystems 7500 machine (ABI, USA). Primer sequences were as follows: *IL-6* (forward) 5′-CCAAGAGGTGAGTGCTTCCC-3′ and (reverse) 5′-CTGTTGTTCAGACTCTCTCCCT-3′, *TNF-α* (forward) 5′-GGTGCTCAAGGGCTACGACT-3′ and (reverse) 5′-GACTGTGGTTACCGTCATGGC-3′, IL-1*β* (forward) 5′-GCAACTGTTCCTGAACTCAACT-3′ and (reverse) 5′-ATCTTTTGGGGTCCGTCAACT)-3′, *iNOS* (forward) 5′-GTTCTCAGCC CAACAATACAAGA-3′ and (reverse) 5′-GTGGACGGGTCGATGTCAC-3′, *ROCK* (forward) 5′-AGCTTGTGGTAAGACATGCTTG-3′ and (reverse) 5′-GGGCATCCAATCCATCCAGC-3′, and *RhoA* (forward) 5′-GCAACTGTTCCTGAACTCAACT-3′ and (reverse) 5′-GTGTCCCATAAAGCCAACTCTAC-3′.

### 2.7. Western Blotting

RIPA Lysis Buffer was used to extract cell proteins. Gel electrophoresis was performed, and proteins were transferred to the PVDF membrane (Millipore USA). Then, the membrane was blocked for 2 h at room temperature and incubated with 1 ∶ 1000 GAPDH, iNOS, IL-6, RhoA, ROCK1, ROCK2, NF-*κ*B, I*κ*B, and phosphorylated-I*κ*B antibodies at 4°C overnight. Subsequently, HRP-conjugated Goat anti-rabbit antibody (1 : 10000) was added and incubated for 2 h at room temperature. The membrane was detected with ECL buffer (Thermo Fisher Scientific, USA) by the Chemiluminescence imager (Tanon, China). Protein levels were normalized to GAPDH. The expression of phospho-I*κ*B was measured by the ratio of phospho-I*κ*B to total I*κ*B.

### 2.8. Statistical Analysis

The experimental results were expressed as means ± SD. The SPSS 20.0 software was used to compare the differences between groups. Statistical differences among groups were analyzed by one-way ANOVA or two-tailed Student's test. The differences were considered statistically significant with *P* < 0.05.

The article "Mechanical Stretch Promotes Macrophage Polarization and Inflammation via the RhoA-ROCK/NF-κB Pathway" was published in 2022. Journal: Biomed Res Int.

## 3. Results

### 3.1. RAW264.7 Cell Morphological Changes after Mechanical Stretch

RAW264.7 cells were mechanically stimulated using the Flexcell-5000T stretch culture system for 8 h at 5, 10, and 15% elongation, respectively (Figure 1(a)). Microscopic observation revealed extended tentacles and irregular growth (Figure 1(b)). Observation of the cytoskeleton by FITC-phalloidin fluorescence staining also revealed that, compared with the control group, the cytoskeleton lost its rounded state after mechanical stretch and presented a polygonal shape, with elongated cell and irregular barbs (Figure 1(c)).

### 3.2. Mechanical Stretch Increased Proinflammatory Cytokine Secretion in RAW264.7 Cells

To determine the effect of mechanical stretch on macrophage, the expression of proinflammatory factors TNF-*α*, iNOS, IL-1, and IL-6 was investigated. As shown in Figure 2(a), culture supernatants after stimulation were collected for cytokine detection using ELISA. The levels of secreted cytokines TNF-*α*, iNOS, IL-1, and IL-6 were increased in the stretched cells positively correlated with elongation compared to nonstretched control. Meanwhile, after mechanical stretch, mRNA expressions of TNF-*α*, iNOS, IL-1, and IL-6 were significantly increased (Figure 2(b)). Taken together, these data showed that mechanical stretch can upregulate the production of proinflammatory cytokines in RAW264.7 macrophages (*P* < 0.05, Figure 2).

### 3.3. Mechanical Stretch Promoted the Expression of the ROCK1, ROCK2, and RhoA in RAW264.7 Cells

RhoA and its downstream effector ROCK regulate multiple cellular processes such as cell morphology and cytoskeleton regulation and play an important role in the response and conduction of extracellular mechanical stimulation. So, we measured the protein expression of RhoA, ROCK1, and ROCK2 in MS-treated RAW264.7 cells. Notably, expressions of ROCK1, ROCK2, and RhoA were significantly increased compared with the control group. These results indicate that mechanical stretch promotes the expression of proinflammatory cytokines, which is related to the activation of RhoA-ROCK signaling pathway (*P* < 0.05, Figure 3).

### 3.4. Mechanical Stretch Increased the Ratio of CD11b+CD86+ Cell Subsets in RAW264.7 Cells

Macrophage polarization is related with inflammatory response. To verify the regulatory effect of mechanical stimuli on macrophage activation, CD11b+, CD206+, and CD86+ cell subsets in RAW264.7 cells were analyzed by FCM. Our data suggested that the proportion of CD11b+CD86+ subsets and CD11b+CD206+ subsets was increased significantly in the MS group positively correlated with elongation compared with the control group, and in particular, the levels of CD11b+CD86+ subsets were much higher. Remarkably, we found that in cells treated with Y-27632, the proportion of CD11b+CD86+ subsets of RAW264.7 cells in the MS group was significantly reduced compared with that of the MS group without Y-27632. However, interestingly, there was much more CD11b+CD206+ cells in the Y-27632 treated MS group compared with the MS group without Y-27632. The results showed that mechanical stretch increased the M1 and M2 type macrophage polarization of RAW264.7 cells. The inhibition of ROCK signal by Y-27632 can downregulate M1-type polarization and promote M2-type polarizations (*P* < 0.05, Figures 4 and 5).

The article "Mechanical Stretch Promotes Macrophage Polarization and Inflammation via the RhoA-ROCK/NF-κB Pathway" was published in 2022. Journal: Biomed Res Int.

### 3.5. Mechanical Stretch Increased NF-*κ*B Activation through Upregulation of RhoA-ROCK Signal in RAW264.7 Cells

Several studies have shown that NF-*κ*B signaling pathway plays an important role in mediating macrophage M1 polarization and inducing inflammatory genes. In the current study, the protein expressions of NF-*κ*B p65, p-I*κ*b-*α*, and I*κ*b-*α* were significantly increased after mechanical stretch stimulation, as well as the expression of RhoA, ROCK2, and ROCK1 in RAW264.7 cells. Then, we treated the cells with Y-27632, a ROCK inhibitor, for 12 h before stretching. Subsequently, upregulation of NF-*κ*B p65 and ROCK was measured as well. Our results showed that MS-enhanced ROCK1, ROCK2, and NF-*κ*B p65 expression and I*κ*b-*α* phosphorylation were significantly blunted. Meanwhile, these upregulation effects of MS on cytokine secretion were largely inhibited by Y-27632 treatment. These results indicate that the suppression of ROCK can reduce the activation of the NF-*κ*B involved in macrophage polarization, thereby alleviating inflammatory response induced by mechanical stress (*P* < 0.05, Figure 6).

## 4. Discussion

Commonly, appropriate and controlled inflammation protects us from multiple harmful stimuli by removing pathogens. But, exaggerated inflammatory response can result in local tissues and systemic injuries and damages [1]. The M1 macrophages identified by CD86 and their secreted proinflammatory cytokines like IL-6 and TNF-*α* play a vital role in the pathophysiological process of inflammation cascade reaction which contribute to the rapidly progressive development of multiple diseases including osteoarthritis, cancer, cardiovascular, atherosclerosis [4, 8]. And M2 macrophages characterized by CD206 play a significant role in protecting the host by limiting excessive inflammation and promoting tissues repair [4, 10, 11]. In addition to biological and chemical factors, currently, researchers pay more attention to the effect of multiple mechanical microenvironments existing in human body including joints, muscles, or blood vessels on the macrophage behavior [30, 31]. The study of Li et al. [32] showed that the pulmonary mechanical ventilation could cause increased secretion of inflammatory factors through macrophages [33]. The results of Yamamoto et al. [18] suggest that hypertension, a kind of mechanical stress in body, may be involved in the atherogenesis through biomechanical stimulation of vascular macrophages. Pongkitwitoon et al. [16] showed that low-intensity vibrations can reduce the protein expression of proinflammatory factors IL-6 and IFN-*γ*. Sridharan et al. [27] indicated material mechanical stiffness plays an important role in the polarization state, function, and migration mode of macrophages. In this study, we applied a horizontal and transverse mechanical load to stretch RAW264.7 macrophages using the Flexcell-5000T stretch culture system. We found that mechanical stretch can mediate RAW264.7 macrophage polarization and enhance the inflammation in vitro, which is associated with the activation of RhoA-ROCK/NF-*κ*B signal. These findings may develop a novel understanding and a potential therapeutic target for mechanical load participated pathophysiological process of inflammation.

The article "Mechanical Stretch Promotes Macrophage Polarization and Inflammation via the RhoA-ROCK/NF-κB Pathway" was published in 2022. Journal: Biomed Res Int.

Macrophages, as an important component of the innate immune system, perform a variety of immune responses including defense against pathogens and maintenance of tissue homeostasis [34]. Stimulated by chemical, physicochemical, structural, and mechanical cues received from the microenvironment, macrophages activate and polarize to different phenotypes [35]. This study showed that MS significantly increased the secretion of proinflammatory cytokines IL-1, IL-6, TNF-*α*, and iNOS in cellular supernatant of RAW264.7 macrophages and the mRNA expression of these proinflammatory factors, which was highest expressed in cells with 15% elongation. After 8 h of MS stimulation, RAW264.7 macrophages changed into activated morphology that the cells lost their roundness and extended many irregular barb-shaped antennae. Furthermore, our study revealed that MS significantly increased the proportion of CD11b+CD86+ macrophage subpopulation of RAW264.7 macrophages that were positively correlated with elongation. The proportion of CD11b+CD206+ macrophage subpopulation also slightly upregulated in the MS group. These findings showed that mechanical stretch could independently promote activation of macrophages, cause more M1 polarization than M2 polarization in RAW264.7 macrophages, therefore leading to the overwhelming inflammation.

The article "Mechanical Stretch Promotes Macrophage Polarization and Inflammation via the RhoA-ROCK/NF-κB Pathway" was published in 2022. Journal: Biomed Res Int.

In addition, RhoA-ROCK activation in RAW264.7 macrophages was observed after stretch stimulation. RhoA-ROCK is a regulatory factor that regulates the stress fibers of cells and mediates corresponding external mechanical stimulation of cells, causing cell migration, movement, and polarity, gene expression changes, vesicle transport, etc. [36, 37]. Kao et al. [38] found that mechanical pulling can activate RhoA-ROCK protein in smooth muscle cells. The study by Boyle et al. [39] showed that acute compressive stress can disrupt the homeostasis of cancer cells which is closely related to RhoA-ROCK signaling pathway. Nakagawa et al. [40] demonstrated that cyclic stress can stimulate chondrocytes through activation of RhoA-ROCK mediated p38 phosphorylation and matrix metallopeptidase 13 (MMP13) expression. These studies indicate that RhoA-ROCK signaling may play a key role in mechanochemical signal transduction in the intracellular environmental changes caused by mechanical stimulation.

After confirming the activation of the RhoA-ROCK signal, we investigated its downstream effectors. NF-*κ*B is one of the key transcriptional regulators modulating polarization of M1-type macrophages [41]. Stimulated by LPS, toll-like receptor 4 (TLR4), and other external factors, NF-*κ*B activation and nuclear transfer can be triggered by I*κ*b phosphorylation, and the expression of polarization-related genes in M1-type macrophages can be promoted [42]. Our results showed that when RhoA-ROCK signal was activated, the expression of NF-*κ*B signal was upregulated and the level of I*κ*b phosphorylation significantly increased. This was accompanied by the upregulation of M1-polarization-related inflammatory factors IL-1, IL-6, and iNOS. We then verified the relationship between these signaling molecules using the ROCK inhibitor Y-27632. The results showed that inhibition of ROCK downregulated the expression of NF-*κ*B p65 and decreased the phosphorylation level of I*κ*b, subsequently decreased the protein expression of IL-6 and iNOS. ROCK inhibition also significantly reduced the proportion of CD11b+CD86+ cell subset (M1-type) in RAW264.7 macrophages as detected by FCM. Interestingly, RAW264.7 macrophages treated with Y-27632 had significantly higher proportion of CD11b+CD206+ cell subset (M2-type). These results indicated that activation of RhoA-ROCK signal may impede macrophage M2 polarization induced by MS, and we will confirm it in future experimental study. Together, these results suggest that activation of RhoA-ROCK-NF-*κ*B signal pathway may play a crucial role in the process of MS-induced inflammation and macrophage polarization.

## 5. Conclusion

Our study shows that mechanical stretch can regulate RAW264.7 macrophage polarization and enhance the inflammatory response in vitro, which may contribute to the upregulation of RhoA-ROCK/NF-*κ*B pathway. We hope that the insights gained in our study will aid future research on the development and treatment of inflammatory diseases involving macrophages.

The article "Mechanical Stretch Promotes Macrophage Polarization and Inflammation via the RhoA-ROCK/NF-κB Pathway" was published in 2022. Journal: Biomed Res Int.

## 6. Practical Applications

This study investigates the effect of mechanical stretch on macrophages in vitro. These data indicate that intermittent cyclic mechanical stretch can regulate RAW264.7 macrophage polarization and enhance the inflammatory response in vitro, which is associated with the RhoA-ROCK/NF-*κ*B pathway. Our findings contribute to a better understanding of the effects and mechanism of mechanical cues on macrophage function and polarization, which may aid future research on the development and treatment of inflammatory diseases involving macrophages.

## Figures and Tables

**Figure 1:** Mechanical stretch promoted M1-type morphological changes in RAW264.7 macrophages. (a) Schematic of Flexcell-5000T applying mechanical stretch. (b) The morphological changes of RAW264.7 macrophages were observed after 5%, 10%, and 15% elongation mechanical stretch for 8 h. Control indicates cells were cultured at static condition (100x). (c) FITC-phalloidin immunofluorescence staining of cytoskeleton in RAW264.7 macrophages after 5%, 10%, and 15% Elong mechanical stretch for 8 h. Control indicates cells were cultured at static condition. DAPI detected nuclei. The white arrow points to the cell antenna. (400x).

**Figure 2:** Mechanical stretch promoted the expression of M1-related mRNA and cytokine secretion of RAW264.7 macrophages. (a) IL-1*β*, IL-6, TNF-*α*, and iNOS concentration in the cellular supernatant after 5%, 10%, and 15% Elong mechanical stretch for 8 h. Control indicates cells were cultured at static condition. (b) IL-1*β*, IL-6, TNF-*α*, and iNOS mRNA expression levels after 5%, 10%, and 15% elongation mechanical stretch for 8 h. Control indicates cells were cultured at static condition. The results are expressed as the means ± SD (*n* = 3). Compare to control, ^∗^*P* < 0.05 and ^∗∗^*P* < 0.01.

**Figure 3:** Mechanical stretch activates the Rho/ROCK1/NF-*κ*B signaling pathway in RAW264.7 macrophages. Protein expression of GAPDH, RhoA, ROCK1, and ROCK2 was analyzed by Western blotting after 5%, 10%, and 15% elongation mechanical stretch for 8 h. Control indicates cells were cultured at static condition. The results are expressed as the means ± SD (*n* = 3). Compare to control, ^∗^*P* < 0.05 and ^∗∗^*P* < 0.01.

**Figure 4:** Inhibition of ROCK1 signal can downregulate M1-type polarization level of RAW264.7 macrophages. The proportion of CD11b+CD86+ cell subset of RAW264.7 macrophages was analyzed by flow cytometry after 5%, 10%, and 15% Elong mechanical stretch for 8 h. Control indicates cells were cultured at static condition. The (+) Y-27632 group was pretreated with Y-27632 (10 *μ*M, 12 h). Quantitative analysis of the ratio of M1-RAW264.7 macrophages via the IDEA software. The results are expressed as the means ± SD (*n* = 3). Compare to control, ^##^*P* < 0.01. Compare to MS group, ^∗∗^*P* < 0.01.

The article "Mechanical Stretch Promotes Macrophage Polarization and Inflammation via the RhoA-ROCK/NF-κB Pathway" was published in 2022. Journal: Biomed Res Int.

**Figure 5:** Inhibition of ROCK1 signal can upregulate M2-type polarization level of RAW264.7 macrophages. The proportion of CD11b+CD206+ cell subset of RAW264.7 macrophages was analyzed by flow cytometry after 5%, 10%, and 15% Elong mechanical stretch for 8 h. Control indicates cells were cultured at static condition. The (+) Y-27632 group was pretreated with Y-27632 (10 *μ*M, 12 h). Quantitative analysis of the ratio of M2-RAW264.7 macrophages via the IDEA software. The results are expressed as the means ± SD (*n* = 3). Compare to control, ^##^*P* < 0.01. Compare to MS group, ^∗∗^*P* < 0.01.

**Figure 6:** Inhibition of ROCK1 signal can inactivate ROCK1/NF-*κ*B pathway of MS-treated RAW264.7 macrophages. Protein expression of IL6, iNOS, Rho, ROCK1, ROCK2, NF-*κ*B, I*κ*b-*α*, and p-I*κ*b-*α* was analyzed by Western blotting after 5%, 10%, and 15% Elong mechanical stretch for 8 h. Control indicates cells were cultured at static condition. The (+) Y27632 group was pretreated with Y27632 (10 *μ*M, 12 h). Control indicates cells were cultured at static condition. Quantitative analysis of protein via the Image J software. The results are expressed as the means ± SD (*n* = 3). Compare to control in MS, ^∗^*P* < 0.05 and ^∗∗^*P* < 0.01. Compare to control in MS+Y-27632: ^#^*P* < 0.05 and ^##^*P* < 0.01. Compare to MS group, ^∗^*P* < 0.05 and ^∗∗^*P* < 0.01.

## Data Availability

All data generated or analyzed during this study are included in this published article.
